This article has been retracted.

# Silicon fertilization counteracts salinity-induced damages associated with changes in physio-biochemical modulations in spinach

**DOI:** 10.1371/journal.pone.0267939

**Published:** 2022-06-09

**Authors:** Riffat Naz, Qamar uz Zaman, Saba Nazir, Nayab Komal, Yinglong Chen, Kamran Ashraf, Asma A. Al-Huqail, Alanoud Alfagham, Manzer H. Siddiqui, Hayssam M. Ali, Faheema Khan, Khawar Sultan, Quratulain Khosa

**Affiliations:** 1 Department of Environmental Sciences, The University of Lahore, Lahore, Pakistan; 2 The UWA Institute of Agriculture, and School of Agriculture and Environment, The University of Western Australia, Perth, Australia; 3 Institute of Soil and Water Conservation, Chinese Academy of Sciences, and Northwest A&F University, Yangling, China; 4 Department of Food Science and Nutrition, Government College University, Faisalabad Sahiwal Campus, Sahiwal, Pakistan; 5 Department of Botany and Microbiology, College of Science, King Saud University, Riyadh, Saudi Arabia; Bangabandhu Sheikh Mujibur Rahman Agricultural University, BANGLADESH

## Abstract

Plant growth and productivity are limited by the severe impact of salt stress on the fundamental physiological processes. Silicon (Si) supplementation is one of the promising techniques to improve the resilience of plants under salt stress. This study deals with the response of exogenous Si applications (0, 2, 4, and 6 mM) on growth, gaseous exchange, ion homeostasis and antioxidant enzyme activities in spinach grown under saline conditions (150 mM NaCl). Salinity stress markedly reduced the growth, physiological, biochemical, water availability, photosynthesis, enzymatic antioxidants, and ionic status in spinach leaves. Salt stress significantly enhanced leaf Na^+^ contents in spinach plants. Supplementary foliar application of Si (4 mM) alleviated salt toxicity, by modulating the physiological and photosynthetic attributes and decreasing electrolyte leakage, and activities of SOD, POD and CAT. Moreover, Si-induced mitigation of salt stress was due to the depreciation in Na^+^/K^+^ ratio, Na^+^ ion uptake at the surface of spinach roots, and translocation in plant tissues, thereby reducing the Na^+^ ion accumulation. Foliar applied Si (4 mM) ameliorates ionic toxicity by decreasing Na^+^ uptake. Overall, the results illustrate that foliar applied Si induced resistance against salinity stress in spinach by regulating the physiology, antioxidant metabolism, and ionic homeostasis. We advocate that exogenous Si supplementation is a practical approach that will allow spinach plants to recover from salt toxicity.

## Introduction

Humans have at least four basic requirements in life: food, clothing, shelter, and fuel [1]. Hence, an adequate supply of food is a basic need of every individual and for that reason, humans depend on plants either directly or indirectly [2]. Green leafy vegetables are naturally rich sources of nutrients [3, 4]. Spinach has a good source of natural bioactive compounds and dietary nutrients which have antioxidant properties and has a role in preventing aging and other age-related disorders. Due to medicinal and nutrient benefits, spinach is a valued crop cultivated on about 921000 ha of land globally with a production of over 26 million tons. In Asia, about 25 million tons of spinach are produced annually [5, 6]. Due to the greater production potential of available germplasm, there are several factors that lead to the yield gap in spinach production, i.e., poor seed germination, inadequate or poor-quality irrigation water, saline soils, poor cultivation practices, and chemical or fertilizer dosage [7]. The Sustainable Development Goal 2 (SDG 2) established by the United Nations aims to achieve zero hunger by ensuring enhanced nutrition and promoting sustainable agriculture through food security. Sustainable crop production is under potential threat throughout the world due to the salinity caused by natural processes, anthropogenic activities, and climate change [8, 9]. According to an estimate about 20% (45 million ha) of irrigated land, producing 1/3^rd^ of the world’s food, consists of saline soil and the area of agricultural land destroyed by salinization is estimated to be 10 million ha annually in the world. It is also estimated that about 50% of the global arable land will be affected by salinity by 2050 [10–12]. Salinity affects growth, ion homeostasis, imbalance of nutrients, and physiological, chemical, and molecular processes of plants which are directly responsible for plant development [13, 14]. Saline conditions affect the nutrient uptake (Ca, K, Mg) resulting in inferior quality of products due to the enhanced concentration of toxic elements that ultimately result in membrane leakage, metabolic and ionic disturbances in spinach [15–18]. In leafy vegetables, salinity stress enhances bioactive leaf pigments, phenolics, flavonoids, polyphenols, and antioxidant activity [19]. Spinach is considered a salt-sensitive vegetable [20, 21]. Salt crop tolerance is rated by salinity threshold (ECt). The majority of vegetable crops including leafy vegetables have a salinity threshold ≤2.5 dS m^-1^ [22, 23].

Salt tolerance of vegetable crops can be enhanced by applying certain nutrients (e.g., silicon, zinc, boron, potassium) and organic acids (e.g., salicylic acid, humic acid, aspartic acid). The application of biostimulant substances controls abiotic stress and improve the growth of plant by improving physiological, catabolism/anabolism, and molecular reactions [18]. Silicon (Si) is the second most abundant element in the earth’s surface and it accumulates in plant cells [24]. Optimum K⁺/Na⁺ ratio, ionic homeostasis, ROS production, and nutrient balance are maintained by the exogenous application of Si which has also been proven to be an eco-friendly approach. Similarly, another study about maize showed that Si treated plants improved photosynthetic efficiency and enhanced growth and yield attributes as compared to salinity stressed plants [25]. In various previous studies involving Si treatments have shown to improve salinity tolerance in various plants i.e., wheat [26], barley [27], maize [28], sorghum [29], cucumber [30], rice [31], canola [32], tomato [33], and okra [34]. The extent of Si mediated benefits under salinity largely varies from species to species and mostly depends on plant genetic makeup to uptake the element [35]. But there is limited information about the exogeneous application of Si for alleviation of salinity stress in spinach. Therefore, it is interesting to investigate the beneficial role of Si under the salinity stress in spinach plants. This study is, therefore, undertaken to appraise the exogenous impact of Si treatments on plant growth, biomass, physio-biochemical, antioxidant activity, and quality attributes by decreasing deleterious effects of salt stress in spinach plant organs grown in salt-affected soils.

## Materials and methods

### Experimental design and treatments

The pot experiment was carried out in a naturally-lit glasshouse at the Department of Environmental Sciences, The University of Lahore, Pakistan. A completely randomized design (CRD) was used in this study consisting of two factors: salinity levels (0 and 150 mM NaCl) and Si application doses (0, 2 mM, 4 mM and 6 mM) using potassium silicate (K_2_SiO_3_) as a salt with three replications.

### Experiment setup and maintenance

Seeds of a spinach variety (Desi), were used as test cultivars that were obtained from the Ayyub Agricultural Research Institute, Faisalabad, Pakistan. The seeds were sterilized with 0.1% (w/v) sodium dodecyl solution and then washed with deionized water. Plants were grown into plastic pots (top diameter~22.5 cm, base diameter~16.5 cm & depth ~18 cm) having about 7 kg of soil per pot and each containing 10 seeds of spinach. The physico-chemical attributes of the soil are given in (Table 1). The initial salinity of the soil was measured using an EC meter (STARTER 3100). After 10 days of sowing, five healthy plants were selected and maintained in the pots. All pots were placed in an open area under normal environmental conditions awaiting the application of stress treatments of salinity. Tap water was used as a source of irrigation at the field capacity level daily. Hoagland solution (50%) was used as a source of nutrients, applied @ of 1 liter per week per pot. Salinity treatments (150 mM) were prepared with NaCl based on the soil saturation percentage as described by Keshavarzi et al. [36]. After an acclimatization period of 15 days (25 days after sowing), salinity treatment was applied to all plants. A set of plants was treated with distilled water that served as a mock control. To attain the required salinity level of 150 mM NaCl, an aliquot of 50 mM NaCl in Hoagland nutrient medium solution was applied every day to achieve the desired level of salinity. After adding salt solution to soil, the soil EC was measured and it was recorded (9.07 dS m^-1^). The salinity of the soil was maintained in successive three-time intervals to avoid salt injury [37]. After 15 days of complete salt stress, foliar application of Si (2, 4, & 6 mM), was applied as per treatment. Two sprays were employed at 10 days intervals using 500 ml of solution as per treatment as described by Naqve et al. [37]. After 25 days of treatment application (65 days after sowing), data for physiological, biochemical, and related characteristics were recorded. The following observations were documented during the various stages of the investigation.

**Table 1:** Basic physico-chemical attributes of experimental soil.

Soil Attributes	Values (Means ± SE)
Sand (%)	49 ± 2.03
Silt (%)	33 ± 2.19
Clay (%)	18 ± 1.89
Textural Class	Sandy Clay Loam
pH	7.05 ± 0.09
Electrical Conductivity (dSm^-1^)	1.45 ± 0.08
Soluble CO_3_^2-^ (mmol_c_ L^-1^)	0.81 ± 0.01
Organic Matter (%)	0.67 ± 0.12
Saturation Percentage (%)	31 ± 0.08
Total Nitrogen (%)	0.041 ± 0.02
Extractable Potassium (mg kg^-1^)	108 ± 3.12
Available Phosphorous (mg kg^-1^)	3.12 ± 0.09

### Growth attributes

The plants were harvested after 65 days of sowing and separated into leaves and roots to measure the growth parameters. Before being separated into leaves and roots, the number of leaves was counted. Height of plant and the leaf length and width (in cm) were measured using a scale. Leaf area (cm^2^) was measured by multiplying the length and width of the leaf. Plants were then washed with distilled water to remove adhered soil particles and were then air-dried. Fresh weight (g) of root and leaves was then measured using an analytical balance. The roots and leaves were oven-dried at 70°C for 48 h for the estimation of the dry weight of root and leaves, separately.

### Gas exchange attributes

Stomatal conductance (*g*_*s*_), photosynthetic rate (*A*), and transpiration rate (*E*) were measured on fully expanded uppermost leaves with portable IRGA (Infra-Red Gas Analyzer, Hoddesdon, UK) at the light saturation intensity between 9:00 am and 12:00 noon on a sunny day as described by Emanuil et al. [38].

### Biochemical attributes

#### Electrolyte leakage (%)

Small pieces of leaves were dipped in deionized water and the electrolyte leakage (EL) level was measured. The first reading of EL was taken after incubation of the sample at 32°C for 2 h and the second reading was taken after incubation of the sample at 121°C for 20 min [39]. To calculate the EL level of samples following formula was used:

$$EL=(EC_{1}/EC_{2})\times 100$$

#### Chlorophyll contents (mg g^-1^ FW)

A crushed sample of plant leaf (~5g) was added to a test tube containing 85% acetone (v/v) and was placed under dark conditions for 24 h for the pigment extraction. Then the sample was centrifuged for 10 min at 4000×g at 4°C. With the use of a spectrophotometer (Halo DB-20/ DB-20S, UK) at wavelengths of 470, 647, and 664.5 nm, the amount of chlorophyll in the supernatant was measured, following the methods described by Lichtenthaler [40].

### Enzymatic antioxidants

Fresh spinach leaves (1.0 g) were extracted in 50 mM phosphate buffer (pH~ 7.8) and the homogenate was centrifuged at 15,000×g for 10 min, and the supernatant thus obtained was used for assaying enzyme activity. The activity of peroxidase (POD) was measured according to the method described by Velikova et al. [41]. Catalase activity (CAT) was determined following the method presented by Aebi [42]. The superoxide dismutase activity (SOD) was assayed following the procedure presented by Beauchamp and Fridovich [43].

### Water related attributes

The method of Turner & Kramer [44] was used for relative water contents (RWC) determination, and the following formula was used for the calculation:

RWC=[(FW–DW)/(TW–DW)]×100

Where FW = fresh weight, TW = Turgid Weight, and DW = Dry Weight.

### Mineral attributes

By following the protocols of Estefan et al. [45], the concentration of K^+^ and Na^+^ minerals in leaves of spinach plant was determined using the wet digestion technique. To prepare a sample solution, leaf material of 0.5g was digested in 10ml of di-acids (HNO_3_-HClO_4_). It was very well mixed on a hotplate till the fumes of white color were visible. The prepared sample was cooled and 50 ml of distilled water was added for dilution. By using the flame photometer (Sherwood Flame photometer, Model-410; Sherwood Scientifics, Ltd, Cambridge UK), the concentrations of dissolved ions (K^+^ and Na^+^) were determined and the ratio was computed by using the division method in all samples.

### Statistical analysis

Data collected were tested using Fisher’s Analysis of Variance (ANOVA) technique considering the completely randomized design under the factorial arrangement which was used for the significance testing. The Highest Significant Difference (HSD) test (5% probability level) was applied for means comparison where ANOVA indicated significant differences. All statistical computations were performed on Statistix software version 10 and the Principal Component Analysis (PCA) was done using the Minitab 10 software.

## Results

### Growth and biomass attributes

Salinity stress and various levels of foliar-applied Si significantly (*p* ≤ 0.01) affected both growth and biomass attributes of spinach plants grown in saline soil (150 mM NaCl) than those grown under the control conditions. Salinity stress decreased the plant height (19.96%), number of leaves (21.04%), leaf length (24.62%), leaf width (5.30%), leaf area (28.35%), root fresh weight (11.44%), root dry weight (10.00%), leaf fresh weight (22.75%) and leaf dry weight (21.35) as compared to the control. Maximum plant height (28.4 and 25.2 cm), number of leaves (9 and 7.67), leaf length (18.3 and 14.4 cm), leaf width (4.6 and 4.3 cm), leaf area (84.96 and 62.70 cm^2^), root fresh weight (3.81 and 3.45 g), root dry weight (0.42 and 0.38 g), leaf fresh weight (12.23 and 10.69 g) and leaf dry weight (1.35 and 1.18 g) were observed under normal and saline soil conditions respectively, where the foliar application of 4 mM of potassium silicate solution was applied as compared to control. The decreasing trend in terms of plant height for salinity stress was in the order as S_2_ > S_1_ and for the Si levels of foliar application treatments as 4 mM > 2 mM > 6 mM > 0 mM (Figs 1A–1E and 2A–2D).

**Fig 1:** Growth attributes, A) number of leaves per plant; B) plant height; C) leaf width; D) leaf length and E) leaf area of spinach at harvesting stage in response to silicon (0, 2, 4, 6 mM) and salinity (150 mM NaCl) applications. For each parameter, mean data (± SD, n = 3) with different letters indicate a significant difference (*P* < 0.05).

**Fig 2:** Fresh and dry biomass of roots and leaves attributes A) root fresh weight; B) root dry weight; C) leaf fresh weight and D) leaf dry weight of spinach at the harvesting stage in response to silicon (0, 2, 4, 6 mM) and salinity (150 mM NaCl) applications. For each parameter, mean data (± SD, n = 3) with different letters indicate a significant difference (*P* < 0.05).

### Physiological and water related attributes

Analysis of variance depicted that the salinity stress and different levels of Si solutions significantly (*p* ≤ 0.01) affected the physiological and water related attributes of spinach plants grown in salinity spiked soils. The maximum decrease in transpiration rate (9.49%), photosynthetic rate (22.08%), stomatal conductance (9.62%), and relative water contents (9.22%) were observed in the treatment of salinity stress (150 mM NaCl). However, the maximum increase in the transpiration rate (50.91%), photosynthetic rate (146.09%), stomatal conductance (53.93%), and relative water contents (26.15%) were observed where the exogenous application of 4 mM of potassium silicate solution was applied, as compared to the control under saline conditions (Fig 3A–3D).

**Fig 3:** Physiological and water related attribute A) transpiration rate; B) photosynthetic rate; C) stomatal conductance D) relative water contents of spinach at harvesting stage in response to silicon (0, 2, 4, 6 mM) and salinity (150 mM NaCl) applications. For each parameter, mean data (± SD, n = 3) with different letters indicate a significant difference (*P* < 0.05).

### Enzymatic antioxidants and biochemical attributes

Foliar applications of Si showed a significant impact on biochemical and enzymatic attributes of spinach, as compared to the non-Si treatment. For salinity stress, the maximum decrease in chlorophyll contents (22.51%), carotenoid contents (22.52%), and increase in SOD (11.17%), POD (13.08%), CAT (19.92%), and electrolyte leakage (48.94%) were observed where 150 mM NaCl salinity stress was applied in soils, as compared to the control. Maximum improvement in chlorophyll and carotenoid contents and decrease in SOD (58.74%), POD (43.22%), CAT (59.68%), and electrolyte leakage (46.86%) were observed where 4 mM potassium silicate was applied, as compared to the control in salinity spiked soils (Fig 4A–4F).

**Fig 4:** Biochemical and enzymatic antioxidants attributes A) chlorophyll contents; B) carotenoid contents; C) SOD activity; D) POD activity; E) catalase activity and F) electrolyte leakage of spinach at harvesting stage in response to silicon (0, 2, 4, 6 mM) and salinity (150 mM NaCl) applications. For each parameter, mean data (± SD, n = 3) with different letters indicate a significant difference (*P* < 0.05).

### Ionic status in leaves

Salinity stress and different rates of Si significantly affected the sodium (Na) and potassium (K) contents in leaves of spinach plants grown in saline soils. Salinity stress increased the Na contents (259.57%), K contents (1.29%), and sodium to potassium ratio (261.54%) as compared to the control. Maximum Na contents (0.59 and 2.25%), K contents (4.64 and 4.66%), and sodium to potassium ratio (0.19 and 0.79) under the normal and saline soil conditions, respectively, were observed where the foliar application of 0 mM of potassium silicate solution was applied (Fig 5A–5C).

**Fig 5:** Ionic contents in leaves A) sodium contents; B) potassium contents; C) sodium to potassium ratio of spinach at harvesting stage in response to silicon (0, 2, 4, 6 mM) and salinity (150 mM NaCl) applications. For each parameter, mean data (± SD, n = 3) with different letters indicate a significant difference (*P* < 0.05).

### Principle component analysis

The physico-biological parameters form a cluster due to the close association with each other. The first principal component correlated with five of the original variables (RWC, LFW, RFW, CC, LDW and RDW). In the first principal components, studied attributes showed more close association and are located close to the axis line. Another cluster is of enzymatic antioxidants that show some correlation among each other is also located close to the axis line. A few measured parameters such as Na, K, and EL plot away from the two main clusters indicating individual characteristics (Fig 6).

**Fig 6:** Principal component analysis plot showing correlation among studied variables and clusters at different salinity and foliar applied Si levels in spinach. RWC = relative water contents; LFW = leaf fresh weight; RFW = root fresh weight; CC = chlorophyll contents; LDW = leaf dry weight; RDW = root dry weight; SOD = superoxide dismutase activity; POD = peroxidase activity; CAT = catalase activity; EL = electrolyte leakage; Na = Sodium contents in leaves; K = potassium contents in leaves.

## Discussion

Salinity is a major environmental factor preventing plants from their natural potential growth and exerts a major limitation to physiological health [46]. The leafy vegetables which are grown below the concentration of 50 mM NaCl show standard growth and production but above this level the growth and other metabolic activities of the plants are disrupted [47, 48]. Tanveer et al. [49] described several deformations and attributes of growth including length, weight, number, width, wet and dry weight of leaves, roots, stem, and flowers in leafy vegetables, especially in spinach plants that are affected by saline conditions [50–52]. More prominently, the reduction of growth rate in leaf (Fig 7) and root cells as compared to leaves was detected, as the maintenance of osmotic stress is more important for root cells for, they absorb essential minerals and water for plant growth [53, 54].

**Fig 7:** Pictorial view of various management and data collection activities during the course of the study.

Essential minerals, nutrients, ant-oxidative enzymes, physicochemical and biological properties of the cells under saline conditions are also significantly controlled by the application of Si fertilizer [55, 56]. The use of Si fertilizer enhances the transportation rate of ionic salts and decreases the concentration of Na ions in plants as observed in the root cells of mung beans [51].

Plant growth and development are mostly affected by the gas exchange and water uptake related attributes specifically by root-applied saline stress [57, 58]. Salinity directly damages the cell by changing the function and configuration of the plasma membrane [59]. The rate of photosynthesis is reduced due to the inefficient utilization of light in spinach plants and the occurrence of photoinhibition that reduces stomatal conductance [60]. Abiotic stress causes a low transpiration rate to turgidity loss of guard cells [58, 61] in plants. The turgidity loss of guard cells causes stomatal cessation resulting in a reduced availability of CO_2_ which leads to a decreased photosynthetic efficiency [58, 60]. By the use of Si fertilizer, leaves and stem epidermal cells show minimum loss of water by reducing the rate of transpiration [62–64]. Silicon influences water relations in crop plants by inducing the development of a double layer silica cuticle under the epidermis of the leaf which decreases the loss of water through cuticular transpiration. Silicon increases the stress tolerance of crop plants by extracting water from the soil as a result of root elongation and up-regulation of aquaporin genes [65]. There is a multifunctional role of Si that improves the plant physiology under saline conditions and results in reduced Na^+^ influx, up-regulation of the antioxidant resistance system, improves the rate of photosynthesis, and enriches activity of ribulose biphosphate carboxylase [25, 51, 64, 66].

An important criterion for assessment of the plant’s capability to tolerate salinity stress is electrolyte leakage and relative water content [67, 68]. Under the NaCl stress, a decline in RWC might be linked to a reduction in the water potential of the rhizosphere due to salt induction, which lowers the water extraction ability of the plant from soil to aerial parts of plants [69]. Sairam et al. [70] documented similar findings in wheat plants. Under higher levels of salinity, crop plants showed a significant reduction in RWC [71]. Salinity stress significantly reduced the photosynthetic pigments and increased membrane leakage (Fig 8).

**Fig 8:** Schematic mechanism of damages caused by salt stress in spinach plants and the protective role of Si fertilization to counteract these damages. The presence of a high concentration of salt in the growing medium causes oxidative, osmotic, and ionic stresses to plants. Increasing the sodium ions in soil lowers the soil water potential of plant cells. This reduces water uptake by plants and consequently results in cellular dehydration, biomass reduction ionic imbalance and lipid peroxidation. To combat this issue, plants induce antioxidative pathways. These antioxidants result in lowering of cellular water potential, membrane leakage and maintain a favorable gradient for water uptake from soil to roots. Si alleviate osmotic stress by influencing the restriction of Na^+^/Cl^−^ uptake via root, improving of the photosynthetic process, maintenance of redox homeostasis, and effective management of essential elements. Si fertilization reinforces the tolerance mechanism of plants to salinity induced oxidative stress.

This rapid breakdown or slow mechanism of chlorophyll content synthesis under saline conditions indicates a reduction of the photo-protection mechanism by decreasing the light absorbance [46, 72]. Salt stress induced the damage of plasma membrane by enhancing the electrolyte leakage [73]. The severity of salt stress progressively enhanced the EL and the tolerance rate of plants against salt stress [74]. Exogenously applied Si protects plants from salt induced membrane damage [75]. Silicon fertilizer also provides strength to the cell membrane of those plants which grow under salt stress [75, 76]. The addition of Si fertilizer in saline soils shows the reduction in electrolytic leakage hence preventing ion leakage from the plasma membrane and a decrease in lipid peroxidation [77]. This implies that the Si potentially has an anti-salt stress effect by attaining the stabilization of the plasma membrane [78]. It has been reported that the Si fertilizer shows protective effects in plants against injury and loss of essential minerals under saline conditions [14, 79].

All the enzymatic antioxidants (SOD, POD & CAT) are frequently considered as the important constituents of antioxidant resistance of the crops [80, 81]. In this study, the alterations of SOD, POD and CAT enzyme activities were examined under normal and saline conditions (Fig 8). In leaves, 150 mM NaC1 treatment increased SOD, POD and CAT activities. Salt stress reduced protein synthesis by activating the antioxidant enzymes [81]. The damage in the cell membrane is also observed by the oxidative damage under the salinity atmosphere [82]. Antioxidant enzymes like SOD, CAT, and POD are regulated by reducing the rate of oxidative damage through the use of Si fertilizer [27, 30, 64, 78]. Additionally, Si fertilizer reduces the effects of salinity and moderates the flow of antioxidant enzymes [83]. The photosynthesis and metabolic activities promote growth rate by the regulation of antioxidant enzymes from the use of Si in rice and wheat shoots [77, 84].

Accessibility to vital nutrients is usually reduced by salt stress [79, 85, 86] in most plants. This study revealed that a minimum concentration of Na^+^ was observed in control, and a maximum concentration was found at a high salinity level (150 mM). These results are consistent with Naveed et al. [87] finding of elevated concentrations of Na^+^ in plant cells and tissues due to an increase in salt stress. The increased level of Na^+^ in various parts of the plant (e.g., leaves) is correlated with soil and root ions of Na^+^ [88, 89]. The saline condition produces a major loss of K^+^, due to an imbalance in the uptake of essential nutrients [89, 90]. Higher K^+^ was found in plants where the foliar application of Si (4 mM) was noticed in both normal and salt-stressed plants. This is due to the use of optimum concentration of Si that limits, the access of Na^+^ to exchange sites resulting in an increase in K^+^ for plant uptake [91, 92]. Silicon can also immobilize Na^+^ in plants due to its high absorption ability. By blocking the transpirational flow through precipitation as SiO_2_ in exodermis and endodermis, Si alleviates salt toxicity. The maintenance of K/Na is improved by potassium uptake by Si nutrition (potassium silicate) which has a stabilizing outcome on the activity of proton pump in salt-treated root tips [93]. Previous studies clearly indicate that there is role of Si in the alleviation of salt stress using potassium silicate. The main reason behind the selection of this salt is that Si is more soluble than K. Similarly, the maintenance of K/Na is improved by potassium uptake due to Si nutrition (potassium silicate), which has a stabilizing outcome on the activity of proton pump in salt-treated root tips [94–96]. Foliar applied Si can be used as chelating agent for the management of toxic salts, particularly sodium (Na^+^) and chloride (Cl^−^) ions [87, 97, 98]. The findings of this study provide an efficient way not only for addressing some nutritional and health challenges but also for improving the incomes of farmers in areas affected by salinity. The present investigation is a practical approach to mitigating salinity stress. However, the current investigation’s outcomes are required to be approved in field appraisal and the economic feasibility must also be calculated.

## Conclusions

Salinity stress significantly affected the growth, physiological, water relations, and ionic attributes of spinach plants. Silicon supplementation provided higher growth, physio-biochemical, photosynthetic, and tissue water ionic status under salinity stress conditions as compared to those without Si treatment. Si applications enhanced growth most likely due to the decreased electrolyte leakage. The Si applications in spinach also increased the enzymatic antioxidants. The Na^+^/K^+^ ratio in spinach leaves reduced significantly due to the application of Si in both normal and salinity stressed soils, which could be related to the limited uptake of Na^+^ ions. Treatment with the application of 4 mM Si concentration was found to be the most suitable level in alleviating the salinity-related stress. Moreover, an exogenous application of Si is the environmentally friendly approach for growing spinach under saline conditions. In the future, research activities focusing on specific aspects such as root architecture traits, molecular forms of Si and salinity interactions, economic benefits and diet diversity in addition to vital nutrients, will be the essential agricultural strategies aiming at improving crop yield under abiotic stress.
